The article "Research on Key Technologies of Personalized Intervention for Chronic Diseases Based on Case-Based Reasoning" was published in 2021. Journal: Comput Math Methods Med.

# Research on Key Technologies of Personalized Intervention for Chronic Diseases Based on Case-Based Reasoning

**DOI:** 10.1155/2021/8924293

**Published:** 2021-08-12

**Authors:** Lin Zhang, Ping Qi

**Affiliations:** ^1^Institute of Service Computing, Tongling University, Tongling, Anhui 244061, China; ^2^Institute of Robotics Engineering, Anhui Sanlian University, Hefei, Anhui 230000, China

## Abstract

In recent years, with the acceleration of industrialization, urbanization, and aging process, the number of patients with chronic diseases in the world is increasing year by year. In China, the number of chronic diseases has increased tenfold in 10 years. The percentage of the disease burden in the whole society accounts for 79.4%. Chronic diseases have become the top killer for Chinese people's health. However, for chronic diseases, prevention is more important than treatment. It is the best way to keep healthy. Therefore, health intervention is the key to prevent chronic diseases. Especially now, with the spread of COVID-19 pandemic, reducing the times of hospital check-ups and treatments for chronic patients is practically significant for releasing the stress on medical staffs and decreasing the rate of transmission and infection of COVID-19. In this paper, case-based reasoning (CBR) technology is used to assist personalized intervention for chronic diseases, and the key technologies of personalized intervention for chronic diseases based on case-based reasoning are proposed. The case organization, case retrieval, and case retention techniques of CBR technology in chronic disease personalized intervention are designed, and the calculation of interclass dispersion is added to the distribution of feature words, which is used to describe the distribution of feature attributes in different categories of cases. It provides an effective method for the establishment of personalized intervention model for chronic disease.

## 1. Introduction

In recent years, with the acceleration of industrialization, urbanization, and aging process, the number of chronic diseases in China has exploded, which has increased tenfold during the 10 years. There are nearly 300 million people with chronic diseases, 350 million overweight and obese people, 200 million people with hypertension, 100 million with hyperlipidemia, and 92.4 million with diabetes. The death rate of chronic disease has risen to 86.6% of the total death rate of Chinese residents. The percentage of the disease burden in the whole society accounts for 79.4%. In the next 10 years, 80 million Chinese people will die of chronic diseases. Chronic disease has become China's top one killer, and huge medical expenses will also be the heavy burden for individuals, families, and society.

Common chronic diseases mainly include cardiovascular and cerebrovascular diseases, metabolic diseases, and pulmonary diseases, such as hypertension, diabetes, and coronary heart disease. These chronic diseases are characterized by long course of disease, many complications, and long treatment, which have a serious impact on the health and normal life of patients [1]. In fact, for chronic diseases, prevention is better than treatment. Prevention is the best way to keep healthy. As traditional Chinese medicine says, “three parts cure, seven parts raise.” People cannot live forever, but people can gradually enhance the physical fitness and improve the ability of rehabilitation and antiaging through good living habits and later recuperation, so as to achieve the purpose of prolonging life and to improve the quality of life. Therefore, health intervention is the key to prevent and cure chronic diseases. However, health intervention has a high requirement for specialization, and it is difficult for ordinary residents to carry out their own health intervention. Therefore, case-based reasoning technology can be used to assist the personalized intervention of chronic diseases.

Case-based reasoning (CBR) is written in the book Dynamic Memory, which is written by Roger Schank from Yale University in 1982. It is an important knowledge-based problem solving and learning method emerging in the field of artificial intelligence. It can be used to solve the problem that nonprofessionals are difficult to obtain and to express professional knowledge. CBR solves the existing problem through the reuse or modification of the solution of the most similar case by building a rich case base and looks for the most similar cases in the case base. In the problem to solve mechanism, CBR uses the case-based reasoning strategy and imitates the cognitive way of analogy in human decision-making process to solve the unstructured and knowledge poor domain problems effectively [2–11].

The process of case reasoning usually includes four steps: case representation, case retrieval, case reuse and modification, and case evaluation and learning. Among them, case retrieval is the key step of case reasoning. Only by finding similar cases through case retrieval can it be better for case-based reasoning. At present, case retrieval techniques used commonly include nearest neighbor retrieval, knowledge-guided retrieval, inductive reasoning retrieval, neural network retrieval, classification retrieval, rough set retrieval, and fuzzy retrieval. However, this paper does not use common case retrieval methods. Instead, it is based on the characteristics of common chronic disease cases, draws on the concept of TF-IDF (term frequency–inverse document frequency), combines the calculation method of information entropy, and then determines the weight of the case attributes through the calculation of the interclass dispersion distribution to solve the problem of different attribute weights. In addition, the paper finally compares the relative similarity of cases through the simple theorem of cosines, which greatly improves the efficiency of case similarity retrieval.

## 2. Related Research

Through the CBR research for many years, the author has designed a children's common diseases diagnosis method based on case-based reasoning and the elderly health assessment method based on case-based reasoning and has applied for successfully key project of Anhui province natural science foundation of the higher institutions, The Children's Common Diseases Diagnosis Method Based on Case-based Reasoning Research, and the supported project of excellent young talents in colleges and universities in Education Department of Anhui province, The Study of the Elderly Health Assessment Method Based on Case-based Reasoning. In the process of project research, the author not only puts the designed algorithm into practice and develop children's common diseases diagnosis model software to get access to the software copyright (see Annex 1 for the copyright certificate) but also standardizes the algorithm to make it be applied to other fields of case-based reasoning, successfully applies standardized algorithm to urban traffic guidance, and successfully develops the urban road traffic congestion channel decision support system software to get access to the software copyright (see Annex 1 for the copyright certificate) [11].

In the preliminary research results, either the diagnosis of common diseases in children, or the health assessment of the elderly, or the decision-making of urban traffic congestion, the application fields are relatively narrow. Although the software designed can use the concept of TF-IDF and the calculation method of information entropy to build a case model, and determine the similarity of unknown cases, the descriptions of the distribution of different characteristics in different cases are not too ideal. The results are usually based on known case diagnosis or artificial intervention, directly according to the known diagnostic results of similar cases, without human intervention. Therefore, the intelligent ability needs to be improved.

In order to solve the problem of the generality of the case-based reasoning method and the distribution description of characteristic attributes to improve the intelligence of the algorithm application process. The research groups have established the health big data through the questionnaire survey of urban residents' lifestyle and health status and have proposed the general case-based reasoning method to add interclass dispersion calculation through the analysis of the original model and the continuous testing and improvement of the software. This method is not only applicable to most fields of case-based reasoning but also describes the distribution of feature words among different classes, which solves the problem that IDF overamplifies the function of rare words. The authors apply this approach to personalize interventions for chronic diseases. Through the questionnaire survey of residents' lifestyle and health status, the case base of the case-based reasoning model has been established. Through the search of similar cases, the probability of chronic diseases caused by residents' lifestyle is calculated, and suggestions for reasonable adjustment of residents' lifestyle are given based on the diagnosis and treatment protocol of known patients.

## 3. A Framework of Key Technology Models for Personalized Interventions for Chronic Diseases Based on Case-Based Reasoning

Through the questionnaire survey of the lifestyle and health status of patients with chronic diseases, as well as the diagnosis and treatment protocol of patients with chronic diseases, the case database is established. Through the similarity retrieval of the unknown cases, several cases whose similarity meets the ranking requirements, or several cases whose similarity meets the threshold, are found out. Then, through the analysis of the chronic disease diagnosis and treatment protocol of similar cases, the diagnosis and treatment protocol of new cases can be obtained, so as to provide the diagnosis and treatment service for the chronic disease patients or to provide reasonable preventive measures for the potential chronic disease patients, to reduce the number of chronic patients hospitalized for examination and treatment. With the prevalence of COVID-19, this has practical implications for reducing the stress on medical staffs at this particular time and the rate of transmission and infection of COVID-19. The key technology model framework of personalized intervention for chronic diseases based on case-based reasoning is shown as follows in Figure 1.

In the key technology model of personalized intervention for chronic disease based on case-based reasoning, the first cases collected need to have specific diagnosis and treatment protocols or preventive measures. Then, they need to have standardized descriptions. Different eigenvectors are used to describe the different attributes of the case state and treatment protocol. By retrieving case status one by one, several matching cases with the highest similarity with the new case are extracted from the case base. Then, the availability of the new case is calculated through the utilization rate of a diagnosis and treatment protocol of the most similar case to recommend the diagnosis and treatment protocol of the new case.

## 4. Case-Based Reasoning for Individualized Intervention of Chronic Diseases

The method of personalized intervention for chronic diseases based on case-based reasoning mainly includes four key technologies: standardized representation of case knowledge, case similarity retrieval, case reuse, and case personalized intervention.

### 4.1. Case Knowledge Standardized Representation

Before using CBR, the data should be cleaned and collated first. The data structure should be standardized. Various medical institutions have a large amount of medical data. However, due to local and temporal differences, many data are not only scattered but also have differences in storage structure, description of illness and diagnosis scheme, and attribute characteristics, so it is difficult to compare a lot of data on the same platform.

Here, we use Boolean eigenvectors to represent case knowledge. Since data is not all structured data, and different fields have different emphases on data requirements, so we first set up a Boolean attribute statistical diagram, which means that all evaluation indicators are structured and all attributes are broken down into Boolean options.

Take the questionnaire of lifestyle and health status of urban residents as an example, the sex can be divided into male and female, so the attribute “sex” can be made. The attribute option 1 represents male, and the attribute option 0 represents female. Age is continuous numerical data, which can be divided into several optional Boolean options such as “Child,” “Teenager,” “Youth,” “Middle age,” and “Old age” according to age. The daily sleep time has “less than 6 hours,” “6-7 hours,” “7-8 hours,” and “more than 8 hours” options, so it is divided into “Daily sleep (less than 6 hours),” “Daily sleep (6-7 hours),” “Daily sleep (7-8 hours),” and “Daily sleep (more than 8 hours)” several Boolean options. Then, all the options are made into Boolean eigenvectors, and the attribute statistics of the evaluation indicators are obtained based on this, as shown in the following Diagram 1.

According to the attribute statistics table (Table 1), the original case library can be converted into a Boolean case library. Assuming that the original case library is shown in the following Table 2, the corresponding Boolean case library is shown in the following Table 3.

Through the transformation of the case base, we found that the case attributes would increase. Many optional attributes are divided into several normalized Boolean attributes, which are decomposable from the same attribute. In each case, only one of the Boolean attributes can be selected. However, the converted Boolean case base can make the cases into vectors, which is helpful for the contrast of similar cases. Realizing the structure of data is more helpful for data process. Even if different regions and institutions have different descriptions of the cases, the standardized conversion of the cases can become a structured case.

Assuming that the attributes of the original case database are decomposed into *n* Boolean attributes in the attribute statistics table, each Boolean case after transformation can be represented by an *n*-dimensional feature vector *X*, *X* = (*x*_1_, *x*_2_ ⋯ , *x*_*n*_). In this vector, if the Boolean attribute does not appear, *x*_*i*_ = 0, otherwise, *x*_*i*_ = 1.

We can easily find that the weight of each Boolean attribute should be different in a case of eigenvector representation. The fewer times a Boolean attribute has a value of 1 in all cases, the more typical this attribute is in case evaluation, so its weight should be greater when carrying out case similarity retrieval. On the contrary, if a Boolean attribute has a value of 1 in a large number of cases, that is to say, it is difficult to judge the actual situation of the case through this attribute, and then its weight in the process of case similarity retrieval should be small. Therefore, it is not reasonable to set the weight of all the attributes that appear in the case to 1. This is similar to the inverse document frequency (IDF) of information theory.

IDF, simply to say, is that if a keyword *w* appears in *N* pages, the greater the *N* is, the smaller the weight of *w* is, vice versa [12].

Combining with the calculation method of information entropy, namely, the calculation method of information needed to express the uncertainty of information, we can get the formula for calculating the weight of the attribute of the case: *w*_*i*_ = log_2_(*D*/*D*_*i*_), where *D* is the total number of cases in the case base, and *D*_*i*_ is the number of times that the value of attribute *i* is 1 in all cases in the case base.

It is assumed that there are 1000 cases in the case base, among which 489 cases have a “sex” attribute value of 1. There are 489 males among 1000 cases, so the weight of “sex” attribute is log_2_(1000/489) ≈ 1.03. Similarly, if the number of times that attribute *i* and attribute *j* value 1 in the case are 200 and 50, respectively, that is, *D* = 1000, *D*_*i*_ = 200, and *D*_*j*_ = 50, then, the weight of attribute *I* is log_2_(*D*/*D*_*i*_) = log_2_(1000/200) ≈ 2.32, while the weight of attribute *j* is log_2_(*D*/*D*_*j*_) = log_2_(1000/50) ≈ 4.32. By parity of reasoning, we can get the weight of all the evaluation indicators, so we get the attribute statistics table with weights which are shown in the following Table 4:

Thus, the weight vector of the Boolean attribute can be obtained as follows:

(1) $$\begin{array}{c} W={\left(w_{1},w_{2},\cdots \cdots ,w_{i},\cdots \cdots \right)}^{T}={\left(1.03,0.86,\cdots \cdots ,2.32,\cdots \cdots \right)}^{T}. \end{array}$$

And the weighted vector of each case *i* in the Boolean case base is deduced as follows:

(2) $$\begin{array}{c} wi=X\times W=\left(x_{1},x_{2},\cdots \cdots ,x_{n}\right)\times {\left(w_{1},w_{2},\cdots \cdots ,w_{n}\right)}^{T}=\left(1,0,\cdots \cdots ,1,\cdots \cdots \right)\times {\left(1.03,0.86,\cdots \cdots ,2.32,\cdots \cdots \right)}^{T}=\left(1.03,0,\cdots \cdots ,2.32,\cdots \cdots \right). \end{array}$$

Through the calculation method of IDF and information entropy, the case weighted vector obtained shows a good application effect in the allocation of case eigenvalue weight. However, the original intention of introducing IDF is to suppress the negative impact of the meaningless high-frequency attribute in the case. In addition, when the ratio between the total number of cases and the attribute with the value of 1 is large, the role of the low-frequency attribute is highlighted. However, here is a question which should be discussed: Common attributes are not necessarily meaningless. On the contrary, some patients with chronic diseases will have some inherent habits, or physical health indicators will have some inherent changes. These habits and changes often indicate that people with these habits or changes will suffer from a chronic disease precursor. In the same way, the occasional presence of low-frequency attributes will be treated as high-weight keywords, which will overamplify the importance of these attributes. Moreover, due to the differences of climate, environment, region, living habits, age, sex, and other factors, different categories of people in different regions will lead to the difference in the prevalence of different chronic diseases. In view of these deficiencies, the frequency of occurrence of the *i*th attribute in different classes will directly affect whether this attribute can become the characteristic attribute of the case. Therefore, an item can be added between the original cases to represent the distribution of feature attributes among different classes, that is to say, the interclass dispersion of feature attribute distribution.

The so-called interclass dispersion is the description of the distribution of characteristics attributed in different categories of cases. The characteristic attributes centrally distributed in a certain type of case often have a strong ability to distinguish categories. It is assumed that all cases can be divided into n categories, and *f* (*i*) represents the frequency of occurrence of feature attribute *i* in a certain category of cases, while $\bar{f\left(i\right)}$ represents the average frequency of occurrence of feature *I* in all types of cases.

(3) $$\begin{array}{c} \bar{f\left(i\right)}=\frac{1}{n}\overset{n}{\underset{k=1}{\sum }}f_{k}\left(i\right). \end{array}$$

The overall interclass dispersion is

(4) $$\begin{array}{c} D\left(i\right)=\frac{\sqrt{1/n-1\sum_{k=1}^{n}{\left(f_{k}\left(i\right)-\bar{f\left(i\right)}\right)}^{2}}}{\bar{f\left(i\right)}}. \end{array}$$

Substitute (3) into (4) to get:

(5) $$\begin{array}{c} D\left(i\right)=\frac{\sqrt{1/n-1\sum_{k=1}^{n}{\left(f_{k}\left(i\right)-1/n\sum_{k=1}^{n}f_{k}\left(i\right)\right)}^{2}}}{\bar{1/n\sum_{k=1}^{n}f_{k}\left(i\right)}}. \end{array}$$

Combine the main idea of weight calculation before, if the feature attribute in Formula (5) only appears in a certain type of case, it has the strongest classification ability, so *D*(*i*) is 1. If the frequency of the feature attribute appearing in each category of cases is equal, it is considered that the feature does not have the classification ability. Therefore, *D*(*i*) is 0, and the feature is useless and can be discarded. Thus, the value of *D*(*i*) is between [0,1]. After considered the dispersion between classes, the weight calculation is as follows:

(6) $$\begin{array}{c} w_{i}=\left(\log_{2}\frac{D}{D_{i}}\right)*\left(\frac{\sqrt{1/n-1\sum_{k=1}^{n}{\left(f_{k}\left(i\right)-1/n\sum_{k=1}^{n}f_{k}\left(i\right)\right)}^{2}}}{\bar{1/n\sum_{k=1}^{n}f_{k}\left(i\right)}}\right). \end{array}$$

Although the discreteness between classes is considered here, if the distribution of attributes with two features is basically similar in the same class case, we still cannot accurately judge the distribution of the two fault features. Therefore, we define the information entropy within the same kind of cases, so as to reflect the distribution of feature attributes within the same kind of cases. If the distribution of some feature attribute *i* in a similar case is more uniform, the information entropy in this kind of case is larger, and the feature attribute *i* can more easily reflect the feature information of this kind of case. The calculation formula of the information entropy of a case within the class is

(7) $$\begin{array}{c} E\left(t,C_{k}\right)=-\overset{D}{\underset{j}{\sum }}\frac{{Nd}_{j}}{{NC}_{k}}\mathrm{lg}\frac{{Nd}_{j}}{{NC}_{k}}, \end{array}$$

wherein *Nd* represents the frequency of occurrence of the *j*th value (0 or 1) of feature attribute *i* in class CK cases, and *NC*_*k*_ represents the total frequency of occurrence of feature attribute *I* in class *C*_*k*_ cases.

Finally, based on the interclass dispersion and intraclass information entropy, a relatively accurate calculation method to determine the weight of feature attributes is obtained for the calculation of case class differentiation:

(8) $$\begin{array}{c} w_{i}=\left(\log_{2}\frac{D}{D_{i}}\right)*\left(\frac{\sqrt{1/n-1\sum_{k=1}^{n}{\left(f_{k}\left(i\right)-1/n\sum_{k=1}^{n}f_{k}\left(i\right)\right)}^{2}}}{\bar{1/n\sum_{k=1}^{n}f_{k}\left(i\right)}}\right)*\left(-\overset{D}{\underset{j}{\sum }}\frac{{Nd}_{j}}{{NC}_{k}}\mathrm{lg}\frac{{Nd}_{j}}{{NC}_{k}}\right). \end{array}$$

According to Formula (8), the improved weight algorithm can be used to select the feature attributes, to calculate the weight of each feature attribute, and then to select the *N* cases with the largest weight as the feature vectors of CBR.

### 4.2. Case Similarity Retrieval

Case similarity retrieval is the core of CBR, which aims to retrieve as few approximate similar cases as possible from a large number of cases, as the reference to the solution of the current problem. Common case search strategies include template search strategy, literature search strategy, inductive index strategy, knowledge guide strategy, and nearest neighbor strategy. In this paper, the nearest neighbor strategy is used for case retrieval, but the calculation of similarity is determined by the law of cosines instead of Euclidean distance.

In the knowledge representation of the case, since we have established an attribute eigenvector for each case, we can calculate the size of the angle between two eigenvectors by using the cosine theorem. Since the weights of all indicators are positive, the cosine value between the two eigenvectors is between 0 and 1. The closer the cosine value between two eigenvectors is to 1, the smaller the angle between the two vectors is. It means that the closer the two eigenvectors are to each other. On the contrary, the closer the cosine value between the eigenvectors is to 0, the greater the angle between the two eigenvectors is. It means that the two eigenvectors represent less correlation between the cases.

We know that the cosine of △ABC is cos*A* = *b*^2^ + *c*^2^ − *a*^2^/2*bc*.

At this point, if *b* and *c* are regarded as two vectors starting from *A*, the above formula can be equivalent to cos*A* = 〈*b*, *c*〉/|*b*| · |*c*|, where <*b*, *c*> said vector inner product, and ∣*b*∣ and ∣*c*∣ has said the length of the vector.

Suppose the eigenvectors of the Boolean attributes of case *X* are (*x*_1_, *x*_2_ ⋯ , *x*_*n*_), where *xi* is 0 or 1, and the attribute weight vector *Y* = (*y*_1_, *y*_2_ ⋯ ,*y*_*n*_)^*T*^, then, its weighted eigenvector is (*x*_1_, *x*_2_ ⋯ ⋯, *x*_*n*_) ⋯ (*y*_1_, *y*_2_, ⋯,*y*_*n*_)^*T*^ = (*x*_1_*y*_1_, *x*_2_*y*_2_, ⋯, *x*_*n*_*y*_*n*_).

Therefore, if we assume that the weighted eigenvectors of two cases A and B are (*a*_1_, *a*_2_ ⋯ ⋯, *a*_*n*_) and (*b*_1_, *b*_2_, ⋯, *b*_*n*_), then, the cosine of the angle between them is $\cos\theta =a_{1}b_{1}+a_{2}b_{2}+\cdots \cdots +{\text{a}}_{n}b_{n}/\sqrt{a_{1}^{2}+a_{2}^{2}+\cdots \cdots +a_{n}^{2}}\sqrt{b_{1}^{2}+b_{2}^{2}+\cdots \cdots +b_{n}^{2}}$.

The smaller cos*θ* value of the two vectors is, the smaller the approximation degree of the case will be. On the contrary, the larger cos*θ* value is, the closer the two cases will be. When cos*θ* = 1, the two vectors will completely overlap, that is to say, the attribute indexes of the two cases will be exactly the same.

Therefore, we use the vector angle calculated by the law of cosines to express the similarity of two vectors. For example, if the result of two vectors calculated by the law of cosines is 0.5, then we reckon that the similarity of the two vectors is 50%. Although the nonlinear cosine function is not very accurate to calculate the similarity of the cases, but here, we do not need to calculate the accurate similarity between the cases to be evaluated and each case in the case library, but to know the relative similarity between the cases to be evaluated and the cases in the case library. That is to say, we only need to know which cases in the case library are more similar to the case to be evaluated. Therefore, using the law of cosines to evaluate similarity is simple, which can obtain a good result of corresponding approximation judgment.

### 4.3. Case Reuse and Case Personalized Intervention

Through the Boolean attribute feature vector expression of the above cases and the case similarity retrieval method calculated by the law of cosines, as well as the method of setting a threshold or setting the number of similar cases, a certain number of cases that are most similar to the current case can be obtained, such as setting search for cases where the similarity is over 90%, or search for the top 50 cases with similarity, etc. By obtaining chronic disease diagnosis and treatment plans of similar cases, we can obtain personalized intervention methods for the diagnosis and treatment of new chronic disease patients.

In the process of case similarity retrieval, if we can find cases with a similarity of 100%, we will find exactly the same cases. Then, we can directly reuse the diagnosis and treatment scheme of the case, otherwise.

First of all, we standardize the diagnosis and treatment protocols of all chronic disease cases in the case base and convert the diagnosis and treatment protocols of all cases into Boolean options after comprehensive conversion. This transformation is consistent with the standardized conversion method of cases in the process of case similarity retrieval. When a certain diagnosis and treatment scheme is adopted in a case, it means that the Boolean option value of the scheme is 1; otherwise, it is 0.

After the standardization of diagnosis and treatment schemes, the personalized intervention of diagnosis and treatment schemes in unknown cases are carried out according to the similarity of similar cases CR_*i*_ and the application degree of a diagnosis and treatment scheme CT_*i*_ in all selected cases. Then, the optional rate of diagnosis and treatment schemes in article *j*th of unknown cases is

(9) $$\begin{array}{c} \text{New}\left({\text{CT}}_{j}\right)=\frac{\sum_{i=1}^{n}\left({\text{CR}}_{i}*{\text{CT}}_{j}\right)}{\sum_{i=1}^{n}{\text{CR}}_{i}}*100\%. \end{array}$$

Suppose, in the case base, *N* optional Boolean diagnosis and treatment protocols can be obtained after the comprehensive and decomposed treatment plans of all cases. Through case search, we find the top 50 cases are the most similar to the current unknown cases. The similarity between similar cases and new cases, as well as the diagnosis and treatment protocol of similar cases, is shown in Table 5.

Then, the probability of the new case adopting the diagnosis and treatment protocol 1 is

(10) $$\begin{array}{c} \frac{98.62\%*1+96.98\%*1+95.33\%*1+\cdots \cdots +89.99\%*0+88.73\%*1}{98.62\%+96.98\%+95.33\%+\cdots \cdots +89.99\%+88.73\%}*100\%=97.30\%. \end{array}$$

The diagnosis and treatment protocol of the new case can be given after the adoption rate of all the diagnosis and treatment protocols of the new case has been calculated, and the threshold value of the case adoption rate has been given through manual intervention.

For example, after manual intervention, the adoption rate of diagnosis and treatment protocol in new cases is more than 95%, and these plans can be regarded as the necessary treatment plan. The adoption rate of diagnosis and treatment protocol in new cases is between 75% and 95%, which can be regarded as the optional treatment plan. The adoption rate of diagnosis and treatment protocol in new cases is between 60% and 75%, as reference treatment plan.

In the process of personalized case intervention, in addition to providing case auxiliary diagnosis and treatment information, it can also be used to expand the case base. In the process of case similarity retrieval, if the similarity between the new case and the cases in the case base is lower than a certain threshold (for example, the similarity is lower than 95%), the auxiliary diagnosis and treatment scheme of the new case will be added to the case base as a case after manual intervention.

## 5. Conclusion

This paper puts forward the method of personalized intervention for chronic disease based on case-based reasoning and gives several key techniques in the process of intervention. This algorithm model can be used in the prevention of chronic diseases and also in the auxiliary diagnosis and treatment of chronic diseases. The main idea is to prevent or treat unknown cases through the judgment of case similarity and the diagnosis and treatment scheme of similar cases. In people's daily life, diseases are inevitable. In addition, different medical staff may give different results in the process of disease diagnosis. At this point, diagnosis and treatment experience is particularly important. Patients are more inclined to the diagnosis and treatment plan given by the medical staff with rich diagnosis and treatment experience. We are not saying that experience is always right, but in the case of ambiguity, the experience will be an important reference. The algorithm proposed in this paper is to integrate the experience of different medical institutions and medical staff and then to be applied. Therefore, the algorithm proposed in this paper can not only be used for personalized intervention for chronic diseases but also for personalized intervention for other diseases, even used in other fields. The premise is that the corresponding accurate case base can be established.

The accuracy of the algorithm proposed in this paper depends on the construction of the case base. The richer the cases in the case base are and the more accurate the diagnosis and treatment scheme in the case base is, the higher the feasibility of the auxiliary diagnosis and treatment scheme finally obtained by the algorithm will be. Of course, there are some problems with the algorithm itself:

Second, when the eigenvector is used to represent knowledge, many attributes in the Boolean case base are decomposed from the same attribute in the original case base, which leads to the fact that the eigenvector used is usually a sparse vector. In addition, the thresholds mentioned in case reuse and personalized intervention techniques need to be set by professionals. The manual intervention of professionals is necessary when new cases are added to the case base, which will undoubtedly increase the degree of manual intervention. Therefore, in practical application, how to simplify the existing algorithm by sparse vector algorithm on the basis of ensuring its effectiveness, and how to reduce the degree of manual intervention to improve its working efficiency as far as possible are the directions of future research.

Finally, the effectiveness of the algorithm in the application process is related to the size of the case base. However, with the continuous expansion of the case base, case similarity retrieval will become more and more complex. Therefore, how to improve the efficiency of the algorithm is also one of the future directions.

## Figures and Tables

**Figure 1:** The key technology model framework of personalized intervention for chronic diseases based on case-based reasoning.

**Table 1:** Attribute statistics.

Attribute ID	Attribute content	Attribute description
1	Sex	Male : 1, female : 0
2	Child	Under the age of 12
3	Teenager	Age between 12 and 18
……	……	……
*i*	Daily sleep (less than 6 hours)	/
……	……	……
*j*	Eat fruit per week (more than 1000 g)	/
……	……	……
*k*	Does anyone in the immediate family have diabetes	Yes : 1, no : 0
……	……	……

**Table 2:** Original case library.

ID	Name	Sex	Age	……	Daily sleep	……	Eat fruit per week	……	Does anyone in the immediate family have diabetes
1	Zhang San	Male	65	……	Less than 6 hours	……	250 g-1000 g	……	No
……	……	……	……	……	……	……	……	……	……

**Table 3:** Original case library.

ID	Name	Sex	Child	……	Old age	Daily sleep (less than 6 hours)	……	Eat fruit per week (250 g-1000 g)	……	Does anyone in the immediate family have diabetes
1	Zhang San	1	0	……	1	1	……	1	……	0
……	……	……	……	……		……	……	……	……	……

**Table 4:** Attribute statistics with weights.

Attribute ID	Attribute content	Attribute description	The weight
1	Sex	Male : 1, female : 0	1.03
2	Child	Under the age of 12	0.86
3	Teenager	Age between 12 and 18	
……	……	……	……
*i*	Daily sleep (less than 6 hours)	/	2.32.
……	……	……	……
*j*	Eat fruit per week (more than 1000 g)	/	4.32
……	……	……	……
*k*	Does anyone in the immediate family have diabetes	Yes : 1, no : 0	0.32
……	……	……	……

**Table 5:** Diagnosis and treatment of similar cases.

Case ID	Similarity	Diagnosis and treatment protocol 1	Diagnosis and treatment protocol 2	Diagnosis and treatment protocol 3	……	Diagnosis and treatment protocol *n*
798	98.62%	1	0	1	……	1
1103	96.98%	1	1	1	……	0
6	95.33%	1	0	0	……	1
235	93.75%	1	0	0	……	1
……	……	……	……	……	……	……
39	89.99%	0	0	1	……	1
1295	88.73%	1	1	1	……	0

## Data Availability

The experiment data supporting this experiment analysis are from previously reported studies, which have been cited, and are also included within the article.

## References

[1] Ping C. (2018). Discussion on the intervention effect of individualized community chronic disease management. *Medicine and health care*.

[2] Ji-qiong L., Xing-guo L., Dong-xiao G., Shuai F. (2010). Case based reasoning ISP knowledge reuse method. *Computer Engineering*.

[3] Li L. I., Xiao-zhong F. A., Quan Q., Xiao-ming L. I. (2011). Ontology- based question expansion for question similarity calculation. *Journal of Beijing Institute of Technology*.

[4] Min H., Shen L.-h. (2012). Case-based resoning based on FCM and neural network. *Control and Decision*.

[5] Abdelwahed M. F., Mohamed A. E., Saleh M. A. (2020). Machine learning; findings from Helwan University broaden understanding of machine learning (solving the motion planning problem using learning experience through case-based reasoning and machine learning algorithms). *Journal of Engineering*.

[6] Zia A., Boumans R. (2020). *Designing Participatory Decision Support Systems: Towards Meta-Decision Making Analytics in Then Generation of Ecological Economics*.

[7] Benamina M., Atmani B., Benbelkacem S., Mansoul A. (2019). *Fuzzy Adaptation of Surveillance Plans of Patients with Diabetes*.

[8] Zhang H. (2018). *Research on Case-Based Reasoning for Urban Road Traffic Congestion Safety Decision Support Technology*.

[9] Lin Z., Zhang D. (2016). A novel diagnosis method for paediatric common disease using case-based reasoning. *International Journal of Simulation Systems, Science & Technology*.

[10] Yuguang N., Junjie K., Fengqiang L., Weichun G., Guiping Z. (2020). Science-automation science; researchers at North China Electric Power University detail findings in automation science (case-based reasoning based on grey-relational theory for the optimization of boiler combustion systems). *Energy Weekly News*.

[11] Lin Z. (2021). Research on case reasoning method based on TF-IDF. *International Journal of System Assurance Engineering and Management*.

[12] Jun W. (2012). *The Beauty of Mathematics*.

